This article has been retracted.

# Relating Sustainable Business Development Practices and Information Management in Promoting Digital Green Innovation: Evidence From China

**DOI:** 10.3389/fpsyg.2022.930138

**Published:** 2022-06-21

**Authors:** Wen Huang, Ka Yin Chau, Ip Yun Kit, Naila Nureen, Muhammad Irfan, Azer Dilanchiev

**Affiliations:** ^1^School of Management, Northwest University of Political Science and Law, Xi’an, China; ^2^Faculty of Business, City University of Macau, Macao, Macao SAR, China; ^3^Faculty of International Tourism and Management, City University of Macau, Macao, Macao SAR, China; ^4^School of Economics and Management, North China Electric Power University, Beijing, China; ^5^School of Management and Economics, Beijing Institute of Technology, Beijing, China; ^6^Center for Energy and Environmental Policy Research, Beijing Institute of Technology, Beijing, China; ^7^Department of Business Administration, Faculty of Management Sciences, ILMA University, Karachi, Pakistan; ^8^Department of Economics, Faculty of Business and Technologies, International Black Sea University, Tbilisi, Georgia

**Keywords:** knowledge management process, sustainable development practices, digital green innovation, structural equation modeling, China

## Abstract

Digital green innovations are being implemented in manufacturing to help organizations achieve sustainability by adopting sustainable development practices (SDPC). However, little is known about the impact of the information management process (IMP) on organizations’ digital green innovation. To address this gap, we devised a multidimensional framework based on the resource-based view (RBV) theory that serves as a basis for sculpting how the IMP captured and sustained organizational digital green innovation via SDPCs. 533 respondents from big and medium-sized manufacturing businesses in China were surveyed, and data were analyzed using the structural equation modeling (SEM) approach. The study makes numerous significant findings. *Firstly*, the SDPC’s dimensions (environment, economic, and social) are considerably improved by the IMP’ dimensions (acquisition, dissemination, and application). *Secondly*, SDPC’s dimensions are critical for attaining organizations’ digital green innovation. *Thirdly*, SDPCs’ implementation mediates the linkage between the IMP and organizations’ digital green innovation. Our findings suggest that investing in and implementing cutting-edge technology and sustainable practices are critical for long-term success. Still, soft issues, such as organizational information management, are equally critical in today’s information-based economy. Finally, in light of the study findings, we present theoretical and managerial implications.

## Introduction

The fast use of harmful pollutants connected with the growth of trade and industry has raised strain on the environment and climate (Yang et al., 2021; Fang et al., 2022). Numerous countries have fallen short of meeting the United Nations’ sustainable development goals (SDG) report on environmental performance (Rehman et al., 2020; Islam et al., 2021). Accumulating scientific proof of this proclivity’s detrimental repercussions has raised stakeholders’ pressure on firms to address ecological degradation’s difficulties (Ahmad et al., 2021; Jinru et al., 2021). Such challenges have increased the emphasis on sustainable and green productivity improvements (Wu et al., 2021; Wen et al., 2022) and propagated doubts about the capacity of development components of sustainability to solve such concerns even though boosting long-term competitiveness (Yumei et al., 2021; Irfan et al., 2022).

Ooi (2014) highlighted that firms must understand the importance of the information management process (IMP), considered the most effective instrument for assessing an organization’s competitiveness due to globalization. Darroch (2005) explored that organizations collect, exchange, and use the information to their advantage, as it is considered the primary driver of innovation. The information gathered from different stakeholders enables policymakers to develop a comprehensive strategy for increasing revenue opportunities and assisting them in achieving sustainable and green goals (Irfan and Ahmad, 2021; Irfan and Ahmad, 2022). Abbas and Saǧsan (2019) explored that the IMP allows companies to become accustomed to deviations occurring and enhance operational resilience, therefore assisting the firms in expanding the strategies of green innovation.

According to Yousaf (2021), corporate green innovation (CRGI) garnered considerable study interest recently due to growing ecological issues and shortage of resources. It helps firms produce environmentally responsive goods and procedures, enabling SDG achievement (Rauf et al., 2021; Ahmad et al., 2022). Furthermore, owing to the absence of sustainable and green strategies backed up by well-organized IMP, industrial firms tend to encounter significant barriers to CRGI compliance. IMP is considered the significant component that fosters the implementation of sustainability approaches and impacts CRGI. As a result, the Global Innovation Index (GII) revealed two critical factors impeding innovation: information and invention. An emerging economy like China is regarded as one of the world’s least inventive countries, with an offensive rating. Research on rising economies such as China might help clarify how different IMP-supported techniques can help curb environmental degradation and produce environmentally friendly goods that safeguard the environment and minimize waste materials (Shahzad et al., 2020a).

Shahzad et al. (2021) showed that the primary constraint on innovation in such emerging economies is the lack of an effective IMP in company operations, which is the central focus of this research. It impedes the application of sustainable development practices (SDPC) in manufacturing sectors. Additionally, the application of SDPC is a driving and binding force for green innovation implementation, which may enhance the sustainability of the environment to compete on a global scale via environmental stewardship (Song et al., 2020). Past findings indicate that emerging economies and large enterprises have shifted away from traditional modes of production toward innovative, advanced, and customer-centric modes of production by overhauling and reproducing ecological processes as they have become more involved with their well-being and the environment (Yousaf, 2021). Government and authorities are also much more active in implementing strict rules and regulations governing industrial companies to prevent environmental degradation due to the 2015 Paris Agreement (Irfan et al., 2020).

Numerous scholars have examined the elements affecting CRGI in the manufacturing sector, which is becoming more competitive daily. Several academics have explored external variables affecting an organization’s capacity to support green innovation, including market needs, environmental restrictions, and supplier greening (Shah and Soomro, 2021). Various academics have investigated inner variables affecting CRGI, including the ethical responsibility of corporations, innovation process, and information management framework (Ding et al., 2019). According to Bhutto et al. (2021), information transmission and acquisition are critical components of developing CRGI. Additionally, Shahzad et al. (2020c) discovered that the protection of the environment and sustainability have a beneficial effect on adopting green innovations. Yousaf (2021) indicates that green competencies and practices also significantly impact green innovation.

Additionally, Saunila et al. (2018) discovered that economic, environmental, and social sustainability significantly impact green innovation investment and deployment investments. Nevertheless, SDPC and green policies are still in adolescence (Khan et al., 2021). Detailed research on implementing SDPC for CRGI in emerging economies is urgently needed.

While other scholars have tried to disclose these challenges by utilizing samples from developing and developed countries, China stands out due to various reasons. International and local organizations have recognized the critical nature of SDPCs and technological spillovers to comply with stringent international commerce and investment standards. Thus, the present research focuses on the impacts of IMP on SDPCs to improve China’s CRGI. Scholars have given limited attention to this complicated issue, and no study has been published examining IMP’s influence on SDPC. Additionally, this study aims to give empirical evidence for the influence of SDPC on CRGI. The purpose behind this research is to alleviate the uncertainty around these correlations by combining the research questions of the study, which are stated below:

• What influence does the IMP have on SDPCs and, in turn, on CRGI?
• Do SDPCs act as a buffer between the IMP and CRGI?

The empirical investigation of these research issues contributes to the literature. Firstly, the proposed conceptual framework seeks to determine the degree to which the IMP influences the SDPC and CRGI of firms with an information-intensive point of view through multivariate examination via structural equation modeling (SEM) and qualitative comparative analysis using fuzzy sets. Secondly, this research sheds light on a novel basic idea of businesses’ SDPC that increases CRGI. This research concentrates on SDPC in emerging economies, such as China, where earlier research has been sparse. Additionally, this research helps experts and administrators integrate IMP techniques into business operations, increasing innovation and sustainability. This study highlights the utility of IMP in daily operations and gives insight into how companies may enhance their CRGI. The following section provides theoretical context and a review of the literature. The formulation of hypotheses is discussed in Section “Hypotheses Development.” In Section “Methodology,” the study’s methodology, in Section “Results,” the discussion and findings, and the conclusion and policy implications are discussed in Section “Discussion.”

## Literature Review and Theoretical Framework

### Resource-Based View Theory (RBV)

Numerous research studies over the past decade have concentrated on the internal corporate factor for organizational effectiveness. Barney et al. (2011) highlighted that RBV theory was frequently utilized throughout organizational operations to characterize an organization’s internal capabilities and resources and their link to success and competitiveness. The RBV is a complement theory that may aid in comprehending how an enterprise can maximize particular production/logistical effectiveness by using the greatest equipment and resources (Savino and Shafiq, 2018). According to this notion, organizations acquire a strategic advantage by concentrating on diverse production factors, i.e., tangible and intangible. Such production factors include all tools, skills, technologies, standard operating procedures, expertise and information, characteristics of the organization, and knowledge and information that enable an enterprise to ‘grasp the concept and execute plans that increase its quality and productivity (Barney, 2000).

Additionally, Barney et al. (2011) defined such morphometric elements as VRIN: (a) valuable, (b) rare, (c) inimitable, and (d) non-replaceable. By contrast, Andersén (2021) examined that the RBV is limited to organizational level implications and ignores the influence of SDPCs on green and ecological efficiency. Hert (1995) created a natural RBV in response to this. Additionally, it is argued that the NRBV broadens the scope of RBV by recognizing the relevance of the environment. It may be thought of as a ‘theory of competitive edge depending on the organization’s interaction with the ecological environment.

The natural RBV (NRBV) strives to understand how organizations’ resources and capabilities might result in strategic and environmental advantages. Environmentalists and ecologists have stated that by adopting an NRBV approach, CRGI may boost an enterprise’s prosperity and long-term sustainability (Shahzad et al., 2020a). Nevertheless, it is contingent upon organizations’ enough and critical capabilities and resources (Sarkis et al., 2010). For example, the capacity to continuously develop and adapt industrial activities results in fewer pollutants and expenditures (Hert, 1995), while (Andersén, 2021) explored that a proactive strategic capability results in first-mover advantages at the first level and proactive environmental protection. Likewise, as a driver of economic development, information systems have fostered an information-based vision of the firm (Grant, 1997). A company’s effectiveness is defined by Abbas and Saǧsan (2019) as the capacity of firms to incorporate technical information means that may be leveraged to establish key strengths for green and sustainable performance improvement. In today’s information-based and circular economy, depending on SDPCs and IMP is the optimal strategy for adopting CRGI. It can boost company development by applying natural system redesign and regeneration concepts (Awan et al., 2021). RBV demonstrates that an organization with greater IMP and SDPC seems to have a greater possibility of developing sustainable and green goods. Additionally, a recent study indicates that the IMP, via the SDPC, contributes to developing greener and innovative products with a lower effect on society and the environment, enhancing CRGI.

### Information Management Process

Various companies use “information” to gain an advantage against others to better comprehend and build a competitive strategic plan. Information is formed as a result of interactions between individuals and societal systems; it is described as a collection of coherent ideas that may support the behavior of individuals. According to Ooi (2014), “Information is an insubstantial asset” provides the source of modest advantages to organizations and people due to its difficulty replicating. An earlier study has shown that firms’ ability to develop green innovation requires information from various stakeholders, including vendors, customers, and research centers (Cui et al., 2020). Additionally, Ooi (2014) explored that IMP aids firms in making thoughtful decisions by collecting information through external and internal sources. Various features of the IMP have been used in previous research projects (Abbas and Saǧsan, 2019). We have used three aspects of the IMP in this research: information acquisition (IACQ), information dissemination (IDIS), and information application (IAPP).

According to Ding et al. (2019), IACQ is a critical element of IMP; it enables enterprises to acquire new and updated information from various stakeholders, ensuring continuous improvement in each corporation. In consideration of the changes occurring in the environment of corporates, IACQ enables a complete awareness of all issues, including financial, consumption patterns, and growth of an organization, to ensure continual improvement in the quality of goods and services (Darroch, 2005). Furthermore, it is critical to ensure perfection by empowering staff vigorously in information assimilation (Song et al., 2020). Participation of employees in the information exchange of invaluable information across the organization’s various departments is critical to achieving their intended goals (Awan et al., 2021). Eventually, organizations should acquire information inferred from stakeholders and customers and deliver such information to employees to improve the firm’s operation (Cui et al., 2020). Information-oriented organizations actively encourage employee engagement, which cannot exist without efficiently maintaining the collection, diffusion, and use of pertinent information across several organization departments. Information-based enterprises vigorously encourage employee participation in company affairs and provide suitable recommendations. This is unlikely to happen without meticulous management of the acquiring, allocating, and implementing pertinent information across multiple organization departments.

### Sustainable Development Practices and Corporate Green Innovation

Sustainable development as a contemporaneous technique was established in the early 1990s as a solution provider that connects the environment, social, and economic dimensions of complicated situations at different regional and sectoral levels through various policy measures (Tseng et al., 2018). Such sustainable development tenets are referred to as a triple bottom line (TBL) because they influence current and generations to come (Elkington, 1998). TBL’s strategy uses green and environmentally friendly techniques and technology to create environmentally friendly goods that help mitigate environmental emissions and climate change threats (Tseng et al., 2018). Numerous factors inspire a firm to seek SDPC, including ethical, legal, and economic considerations. Three SDPC elements were chosen for this study: sustainable social practices (SSCP), sustainable economic practices (SECP), and sustainable environmental practices (SENP).

Saunila et al. (2018) highlighted that to minimize environmental degradation, greenhouse effect, and continuous climate change, and we must take a proactive role in commercial disintegration management for environmental stewardship. From the economic standpoint of SDPC, firms that take care to improve environmental sustainability by decreasing unintended consequences of manufacturing operations will also strengthen their economic and financial sustainability. Social elements are primarily concerned with protecting and enhancing the safety and health of external and internal groups, fostering interaction between them, and promoting equality of opportunity and well-being. Wang (2020) explored that with the growing demand for sustainable development, overall organizational standards for competing have been increased to encompass multidisciplinary social, environmental, and economic sustainability practices. The evaluation of such SDPC is considered a means of identifying critical determinants of CRGI.

Corporate green innovation is a notion that is both internally motivated and outwardly responding; it stresses not just originality and the significance of innovation but also resource conservation and the development of environmental sustainability (Ardito et al., 2019). Currently, researchers are emphasizing the competitive edge gained by a company’s sustainable and green activities and its impact on CRGI. Green innovation aims to minimize emissions by producing new goods, services, procedures, and techniques and minimizing the negative environmental consequences of organizations (Abbas, 2020). Additionally, Chen et al. (2006) noted that it is “the primary engine of long-term socioeconomic progress.” CRGI quantifies how firms have enhanced their sustainable product and process innovation over three years.

As a result, Abbas and Saǧsan (2019) validated the concept of CRGI as including both green goods and green process innovation. These initiatives attempt to decrease the use of natural resources, maximize renewable resources, and minimize waste. Manufacturers, particularly, alter the traditional product lifecycle from resource acquisition through product creation, supply chain management, ingestion, and recycling (Awan et al., 2021). Businesses that implemented sustainable dimensions had a tremendous opportunity to acquire new customers. An SDPC is the most effective strategy for increasing innovation that satisfies consumer demands and desires, which is the most critical component for firms seeking to create sustainable and green goods (Ardito et al., 2019).

## Hypotheses Development

### Information Management System and Sustainable Development Practices

#### Information Acquisition

Information acquisition is a term that refers to the process of finding and gaining new information necessary for efficient business operations from a variety of sources, hence improving performance at the individual level and organizational levels (Darroch, 2005). IACQ’s primary objective is to ascertain customers’ requirements and reactions to goods and services. By incorporating a sustainable and green agenda, organizations increase their chances of collaborating and communicating with external stakeholders and gaining access to their newest technology and information (Shah and Soomro, 2021). Scholars have shown a clear correlation between IACQ and organizational performance (Cui et al., 2020). While several academics explored a negative correlation between IACQ and organizational performance, they continue to advocate for R&D investments to generate new ideas to improve innovativeness. Furthermore, IACQ positively influences firm performance (Lee et al., 2013).

Abbas and Saǧsan (2019) opined that firms should use acquired information in their operations to achieve sustainable development objectives. According to Shahzad et al. (2020b), information assimilation has a significant impact on the sustainability of organizations. These researches emphasized the critical significance of information and the function of IACQ in achieving SDPC (economic, social, and environmental). As a result, the following hypotheses are developed:

H1a: IACQ positively influences SENPs.
H1b: IACQ promotes SECPs.
H1c: IACQ positively affects SSCPs.

#### Information Dissemination

Information dissemination collects, distributes, and communicates information among employees to enhance corporate activities (Shahzad et al., 2021). IDIS may take on several aspects, including information sharing and information collecting; sharing refers to proposing information, while collection refers to gathering information among employees and workers (Lee et al., 2013). A clear correlation between information sharing and service performance has been discovered (Mills and Smith, 2011). According to a previous study, it may be the primary social participation and integration method inside a firm, empowering workers to address challenges via support and inventive ideas (Awan et al., 2021).

Song et al. (2020) suggested that firms promote workers’ information behaviors to improve performance results. Additionally, sharing information positively impacts sustainable growth through green management and technology innovation. They also discovered that IDIS has a beneficial effect on long-term business performance. The flow of information within the organization raises the pace of information sharing between departments and various hierarchies; it also increases the chance of long-term improvement (economic, social, and environmental) (Abbas, 2020). As a result, the following hypotheses are developed:

H2a: IDIS positively influences SENPs.
H2b: IDIS significantly influences SECPs.
H2c: IDIS significantly influences SSCPs.

#### Information Application

Information application is considered incorporating previously acquired information into the design and delivery of final goods to improve overall effectiveness and activities (Mills and Smith, 2011). Additionally, it is considered a reaction to information. IAPP is shown when a firm gathers information about its customers’ requests and consumer preferences and responds quickly to enhance organizational operations. It is critical to foster core skills inside organizations to improve their competitiveness. According to Darroch (2005), IAPP is a necessary component of successful technical improvements in performance. It is considered a vital resource that enables firms to maintain success in today’s competitive environment.

Additionally, IAPP enables organizational capability and information transformation into developing products and operations (Mills and Smith, 2011). Through modern, creative, and digital technologies of manufacturing procedures, organizations may make sustainable goods (Bhutto et al., 2021). IAPP has been utilized to help organizations’ sustainability dimensions to ensure greener development results (Abbas and Saǧsan, 2019). Thus, the concrete implementation of information may be transformed from a prospective capability to an energetic and manifested capability that affects firms’ performance (Mills and Smith, 2011). As a result, it is recommended that IAPP should be included in SDPC (economic, social, and environmental). As a result, the following hypotheses are developed:

H3a: IAPP positively influences sustainable environment practices (SENP).
H3b: IAPP positively influences SECPs.
H3c: IAPP positively influences SSCPs.

### Sustainable Development Practices and Corporate Green Innovation

#### Sustainable Environment Practices

According to Saunila et al. (2018), environmental dimensions of sustainability transform production methods to mitigate adverse environmental impacts and reduce waste materials. Businesses must consider using creative and ecological techniques to minimize utilization and degraded conditions (Song et al., 2020). Previous research conducted by Huang and Li (2017) has shown that firms that have integrated ecological plans and sustainability practices into their operations are capable of producing green goods. Proactive measures related to environmental sustainability lead to a rise in green organizational assimilation for minimal environmental impact (Shah and Soomro, 2021).

Additionally, an erstwhile study conducted by Zhang et al. (2020) indicates that environmental preparedness bolsters organizational innovation and competitiveness. The existing research indicates that environmentally sustainable development is a critical component of green innovation investment and deployment. Environmentally concerned organizations force growth and performance (An et al., 2021). Efficient and environmentally friendly businesses can quickly meet the standards necessary to avert environmental degradation (Chang, 2016).

Additionally, Shahzad et al. (2021) have shown a clear correlation between environmental sustainability and green innovation. As a result, environmental motivations and consciousness of eco-friendly actions are critical in today’s business period for green innovation. As a result, the following theory is advanced:

H4a: Sustainable environmental practices significantly influence CRGI.

#### Sustainable Economic Practices

Economic dimensions of sustainability are composed of two distinct perspectives; the first is related to monetary success, while the other is concerned with the community’s welfare. It was extensively investigated after the worldwide economic slump when the hazards of insolvency and bankruptcy were recognized (Geng et al., 2021). Tseng et al. (2018) emphasized that incorporating recycling concepts into overall organizational logistics helps reduce waste and conserves energy, promoting a stable economy. According to recent research conducted by Khan et al. (2021), lowering manufacturing costs has a beneficial effect on green innovation; they further explained that potential savings and reprocessing are the primary drivers of raw material and energy efficiency.

Abbas (2020) demonstrated that corporate social responsibility (CSR) has a considerable impact on a company’s green outcomes in general for the well-being of society. They also stated that green innovation is influenced by stakeholders involved, such as societies and non-governmental organizations. Additionally, past research discovered that business prosperity correlates with green product innovation but had no correlation with green process innovation (Li et al., 2017). Nonetheless, no relationship exists between CRGI. These ambiguous conditions have encouraged researchers to investigate the link; as a result, the following explanation is advanced:

H4b: SECPs have a beneficial effect on CRGI.

#### Sustainable Social Practices

Social dimensions of sustainability are defined as an organization’s environmental efficiency, emphasizing the development of human capital, employment generation, and societal health (Saunila et al., 2018). Green innovation has significantly been strengthened due to internal information and skills, and development activities (Lim et al., 2017). Intellectual capital and environmental education may also influence employees’ attitudes and behaviors toward environmentally friendly acts. For our setting, green innovation may exert its effect via changes in behavior and attitude, most notably by promoting technology adoption for consumption and collaboration (Hojnik and Ruzzier, 2016). Existing research indicates that ecological information affects organizations’ profitability and social assistance.

Nonetheless, intellectual capital and corporate training developments stimulate the green innovation process. Consumers are now willing to pay a premium for efficient and environmentally friendly items to improve effectiveness and revenue growth (Song and Yu, 2018) ecologically. Previous research conducted by Saunila et al. (2018) has shown that the sustainability social component has a favorable effect on the adoption and investment of green innovations. It has been discovered that green innovation is influenced by organizational needs, green customer requirements, intellectual resources, and internal information abilities. As a result, the following theory is advanced:

H4c: Sustainable social practices positively influence CRGI.

#### The Mediating Role of Sustainable Development Practices

The relevance of SDPC has been a central concern for researchers from various disciplines. For instance, Nidumolu et al. (2009) emphasized the critical role of SDPC in advancing green innovation. Additionally, IMP is a critical approach and facilitator for firms looking to improve their innovation capabilities (Darroch, 2005). Ooi (2014) highlighted that to improve results, it must leverage an appropriate corporate strategy and the commitment of senior management. The IMP, SDPC, and CRGI affiliations form when top management demonstrates a commitment and dedication to preventing the destruction of the environment and invests substantial time in acquiring ecologically friendly and sustainable resources to enhance green innovation through effective management of employees’ information and capabilities. In this scenario, information management stresses incorporating intellectual capital and sustainable business strategies to achieve long-term goals (Davenport et al., 2019). Existing research has shown a clear correlation between IMP and CRGI (Song et al., 2020). Darroch (2005) explored the various types of innovation that need a variety of sources and, hence, a variety of IMP strategies. Additionally, erstwhile studies have examined the direct relationship between several sustainability dimensions and CRGI (Abbas and Saǧsan, 2019).

Nevertheless, no research exists in the present literature that examines the mediating effect of SDPC between IMP and CRGI. This study seeks to determine if SDPC operates as a link between IMP and CRGI. According to the earlier studies, SDPCs will mediate the connection between IMP and CRGI in the following hypothesized manner.

H5: Sustainable development practices act as a mediator between the relationship of IMP and CRGI.

The study framework shown in Figure 1 takes into account the research hypotheses.

**FIGURE 1:** Research framework.

## Methodology

### Procedure and Sampling

Chinese cities may be classified into four groups based on their development stages: first, second, third, and fourth-tier. The first group of cities includes the most advanced economically, socially, and culturally. The second group of cities are the provincial capitals and are moderately established. The third group consists of typically moderately developed cities within every domain, whereas the fourth group consists of cities at the provincial stage (Hao et al., 2016). Under such a perspective, we conducted a comprehensive survey questionnaire in ten cities of China between January to March 2022, in which Shanghai, Shenzhen, and Beijing (1st group), Chengdu, Hefei, and Jinan (2nd group), Xiangfan, and Zhongshan (3rd group), Xinmin and Changshu, (4th group) are included.

We conducted a pilot survey on a smaller sample size before performing the study to ensure the accuracy of the questionnaire and can provide descriptive results (Xue et al., 2014). Later, we contact responders personally (Reuter and Schaefer, 2017). Two sections were made for the entire procedure. In first step, the distribution of questionnaires to 900 participants was included, who were supposed to submit them around one month. Each section of the questionnaire was thoroughly explained to them. Following that, respondents returned the questionnaire within the specified time frame. Five hundred thirty-three valid replies were obtained, representing 59.2% of the original sample. According to Westland’s formula, our model requires a minimum sample size of 427 (Westland, 2010). Nevertheless, our actual sample size (533 respondents) is much greater, demonstrating that the sample size is sufficient for empirical research.

### Measures

The research measured latent components using a 7-point Likert scale (1 demonstrated strongly disagree and 7 represented strongly agree). Additionally, the researchers proposed all items of measurement and scales extracted from earlier research and adapted them for the study environment (Shahzad et al., 2021). All constructs used in this study were drawn from previous studies to ensure contextual coherence, which specialists verified.

#### Information Management Process

Darroch (2005) quantified the IMP paradigm using three critical aspects: IACQ, IDIS, and IAPP. IACQ was assessed using a 6-item scale to gather and quantify information and acquisition. Additionally, a 5-item scale was employed to measure information absorption and transmission of information from inside and outside the organization. Additionally, IAPP was quantified by employing a 5-item scale measuring information’s rapid uptake and reaction. We employed the IMP scale that has been extensively utilized in previous research (Abbas and Saǧsan, 2019).

#### Sustainable Development Practices

Saunila et al. (2018) determined the three-dimensional concept of SDPC, including economic, social, and environmental sustainable dimensions. Each component was quantified by employing 4 to 5 elements representing organizational dimensions relating to waste reduction and management, hazard reduction, energy conservation, cost-effectiveness, income production, and society’s safety and health.

#### Corporate Green Innovation

For assessing CRGI, we adopted (Song and Yu, 2018) construct consisting of six items, which quantifies how firms have enhanced their greener process innovation and green product innovation over the previous three years. CRGI may significantly enhance goods or procedures to reduce emissions, recycle, and create greener goods designs for environmentally responsible manufacturing and performance enhancement.

## Results

### Statistical Summary, Correlation, Convergent, and Discriminant Validity

We employed SEM to examine the formulated hypotheses. The statistical analysis was performed using SPSS (version 26) and AMOS (version 26) software. Table 1 reports the statistical summary of the data. To ascertain the relationship among variables, correlation analysis was utilized. Convergent validity was assessed using average variance extracted (AVE) values and item loadings. The results indicate that the AVE values for all constructs were more than 0.50, suggesting that latent variables maintained at least 50% of the variance. The discriminant validity was assessed using the square root of AVE. The results demonstrate discriminant validity, as the square root of the AVE is greater than its correlation with other variables (Tanveer et al., 2021). The maximum shared variance (MSV) values are lower than AVE values for all variables, further validating discriminant validity (see Table 2).

**TABLE 1:** Statistical summary of the data.

Variable	Observations	Items	Mean	SD	Coefficient of variation (CV)
IACQ	533	5	3.307	0.356	0.108
IDIS	533	4	2.771	1.836	0.663
IAPP	533	5	3.324	0.487	0.147
SENP	533	6	3.518	0.807	0.229
SECP	533	7	2.603	0.994	0.382
SSCP	533	7	2.906	1.896	0.652
CRGI	533	4	2.470	0.600	0.243

**TABLE 2:** Correlation, convergent, and discriminant validity findings.

Variable	IACQ	IDIS	IAPP	SENP	SECP	SSCP	CRGI	AVE	MSV
IACQ	**0.711**							0.505	0.114
IDIS	0.266	**0.832**						0.692	0.335
IAPP	0.274	0.453	**0.817**					0.667	0.287
SENP	0.337	0.357	0.536	**0.803**				0.645	0.287
SECP	0.288	0.213	0.146	0.341	0.845			0.715	0.116
SSCP	0.161	0.557	0.451	0.326	0.215	**0.796**		0.633	0.524
CRGI	0.273	0.579	0.512	0.429	0.214	0.724	**0.747**	0.558	0.524

*Bold values represent AVEs’s root square.*

### Reliability and Multicollinearity Findings

Items’ reliability was determined using the values of Cronbach’s alpha. The values were greater than the minimum tolerable value of 0.70, validating the reliability of the data (Nunnally, 1994). The consistency of variables’ items was determined using the composite reliability (CR). The findings indicate that the CR values exceed the permissible minimum of 0.70 (Hair et al., 2017). Table 3 depicts these results. We conducted a linear regression test to examine the possibility of multicollinearity in our model. The findings indicate that the model is free from multicollinearity since the tolerance and variance inflation factor (VIF) values are within the recommended range (Field, 2013).

**TABLE 3:** Factor loadings of measurements model.

Variable	Items	Standard loadings	Cronbach-α	CR
Information acquisition (IACQ)			0.904	0.803
	IACQ 1	0.787		
	IACQ 2	0.816		
	IACQ 3	0.899		
	IACQ 4	0.864		
	IACQ 5	0.856		
Information dissemination (IDIS)			0.838	0.940
	IDIS 1	0.745		
	IDIS 2	0.719		
	IDIS 3	0.785		
	IDIS 4	0.738		
Information application (IAPP)			0.926	0.933
	IAPP 1	0.779		
	IAPP 2	0.811		
	IAPP 3	0.809		
	IAPP 4	0.847		
	IAPP 5	0.728		
Sustainable environmental practices (SENP)			0.904	0.915
	SENP 1	0.825		
	SENP 2	0.742		
	SENP 3	0.750		
	SENP 4	0.886		
	SENP 5	0.903		
	SENP 6	0.692		
Sustainable economic practices (SECP)			0.934	0.926
	SECP 1	0.829		
	SECP 2	0.900		
	SECP 3	0.879		
	SECP 4	0.898		
	SECP 5	0.836		
	SECP 6	0.738		
	SECP 7	0.723		
Sustainable social practices (SSCP)			0.923	0.896
	SSCP 1	0.716		
	SSCP 2	0.868		
	SSCP 3	0.818		
	SSCP 4	0.877		
	SSCP 5	0.797		
	SSCP 6	0.818		
	SSCP 7	0.812		
Corporate green innovation (CRGI)			0.863	0.835
	CRGI 1	0.715		
	CRGI 2	0.735		
	CRGI 3	0.712		
	CRGI 4	0.679		

### Measurement and Structural Model Testing

The quantitative and structural models were estimated explicitly to assure the validity of the findings (Leguina, 2015). To identify the model, this study employed confirmatory factor analysis (CFA). The examination showed that all the linkages are linear because the *f*-value is high. Moreover, to confirm the similarity of data with the study’s structural model, various fitness tests were employed. The given indices of fitness (i.e., CFI = 0.978, NFI = 0.934, IFI = 0.969, TLI = 0.968, GFI = 0.958, RMSEA = 0.036, X2/df = 1.396, and SRMR = 0.031) were found within the threshold value (Lucianetti et al., 2018).

The path diagram of SEM is shown in Figure 2. A positive and significant association (β = 0.04, *p* < 0.05) was established among IACQ–SENP after scheming the demographic factors. Hence, H1a was accepted. The path coefficient of IACQ with SECP (β = 0.09, *p* < 0.1) shows a positive association between IACQ and SECP. Hence, this study accepted H1b. The IACQ path coefficient does not significantly affect SSCP (β = 0.16); consequently, H1c was rejected. In the same vein, IDIS positively affects SENP as the IDIS path coefficient (β = 0.08, *p* < 0.05) indicates a significant and positive relationship with SENP. As a result, this study accepted H2a. The IDIS path coefficient does not significantly affect SECP (β = 0.29). Hence, H2b was rejected. On the flip side, IDIS positively affects SSCP, as the IDIS path coefficient (β = 0.02, *p* < 0.01) states a positive association with SSCP. Accordingly, H2c was accepted. H3a, H3b, and H3c were also accepted, as IAPP significantly influence SENP (β = 0.06, *p* < 0.05), SECP (β = 0.11, *p* < 0.1), and SSCP (β = 0.31, *p* < 0.05). Similarly, H4a was accepted, as SENP positively influence CRGI (β = 0.01, *p* < 0.01). H4b was also accepted, as SECP significantly influence CRGI (β = 0.13, *p* < 0.1). H4c was also accepted, as SSCP significantly influence CRGI (β = 0.03, *p* < 0.01). The mediating effect of SDP is also significant in the relationship between IMP and CRGI (β = 0.16, *p* < 0.05). Hence, hypothesis 5 was accepted. Table 4 illustrates the results of the hypotheses.

**FIGURE 2:** Path diagram of structural equation modeling (SEM). ***p < 0.01, **p < 0.05, *p < 0.1.

**TABLE 4:** Hypotheses’ findings.

Hypotheses	Hypotheses paths	β-value	*f*-value	Result
H1a	IACQ → SENP	0.041**	126.7**	Accepted
H1b	IACQ → SECP	0.093*	167.5*	Accepted
H1c	IACQ → SSCP	0.163	220.4	Rejected
H2a	IDIS → SENP	0.086**	154.4***	Accepted
H2b	IDIS → SECP	0.291	329.5	Rejected
H2c	IDIS → SSCP	0.026***	110.3***	Accepted
H3a	IAPP → SENP	0.065**	137.1**	Accepted
H3b	IAPP → SECP	0.113*	194.7*	Accepted
H3c	IAPP → SSCP	0.310**	357.5**	Accepted
H4a	SENP → CRGI	0.019***	103.6***	Accepted
H4b	SECP → CRGI	0.137*	201.8*	Accepted
H4c	SSCP → CRGI	0.038***	115.8***	Accepted
H5	IMP → SDPC → CRGI	0.167***	224.5***	Accepted
**Analysis of path coefficients (direct effects)**				
IACQ → CRGI		0.193	2.897	Accepted
IDIS → CRGI		0.128	3.187	Accepted
IAPP → CRGI		0.152	4.351	Accepted

***p < 0.01, **p < 0.05, *p < 0.1.

## Discussion

Resource-based view theory has been used in this study to establish a structure for analyzing the multidimensional interaction between IMP, sustainable development dimensions, and CRGI, which has received little attention before. CRGI is rapidly gaining traction as a powerful instrument for SDPC. Firms are increasingly driven to enhance their CRGI via the mitigation and resolution of environmental challenges. On the other side, CRGI may be a problematic, information-intensive endeavor fraught with complications. Our findings indicate that IACQ significantly affects SENP and SECP, supporting H1a and H1b.

Nevertheless, it has a negligible connection with SSCP (β = 0.16), dismissing H1c and corroborating past research (Zhang et al., 2020). Such negligible finding highlights the essence of building an absorbent ability that enables firms to acquire information from various investors and scurry to address social challenges in emerging nations. IDIS has a favorable interaction with SENP and SSCP, supporting H2a and H2c. Nevertheless, it exhibits a negligible connection with SECP (β = 0.29), indicating that H2b is rejected. Recent investigations by Song et al. (2020) further support our findings. Nevertheless, research by Darroch (2005) contradicts our results, stating that reclusive people avoid interacting and sharing information, which is the reason for decreased information exchange among workers in an organization, hence harming SECPs.

Additionally, IAPP positively correlates with all SDPC dimensions, validating H3a–H3c. To enhance SDPC, the company must effectively use previously gained information to increase client pleasure (Nidumolu et al., 2009). Additionally, the conclusions of this study corroborate previous results (Shahzad et al., 2021). IAPP is considered a critical component of the organization’s ability to develop sustainable goods via new technology. SDPC and CRGI are in their infancy in emerging economies such as China. Additionally, regulatory organizations in industrialized nations encourage sustainable practices via fines for excessive emissions and carbon taxes, which both incentivize enterprises and pressurize them to refrain from harmful operations.

Sustainable development practices are widely regarded as essential engines of green innovation, and their implementation will improve sustainability. This analysis demonstrates that all SDPC characteristics contribute significantly to CRGI, similar to previous research conducted by Awan et al. (2021). They explored that SDPC will enhance green innovation by merging new and greener manufacturing technology. According to our results, SECP is the most critical factor affecting CRGI (β = 0.13), followed by SSCP (β = 0.03) and SENP (β = 0.01). Businesses can evaluate their operating impacts on CRGI by measuring the importance of investing in environmental management systems (Hojnik and Ruzzier, 2016). As the need for eco-friendly goods continues to rise, socially responsible firms are increasingly helpful in meeting customer expectations without causing damage to the environment (Tseng et al., 2018). Cost reduction and energy conservation are compelling factors closely tied to SECP, affecting CRGI.

We suggested that CRGI is achieved when SDPC has become a compulsory part of organizations’ information-driven strategies regarding our last hypothesis. The results revealed that SDPC mediates (β = 0.247), thus supporting H5. We also tested each dimension of the IMP towards CRGI; all are significant and provided in Table 1.

## Conclusion and Research Implication

### Conclusion

By analyzing the link between the IMP, SDPC, and CRGI using SEM, this study adds to the growing area of research on sustainable development and green innovation. Our results indicate that all three IMP dimensions (IACQ, IDIS, and IAPP) substantially affect SDPC components (environment, social, and economic). Additionally, all SDPC aspects have a considerable effect on CRGI, demonstrating the importance of expertise in this subject. Moreover, the study’s significant mediating effect has shed light on another addition to this research. These findings showed that information might be used to accomplish an organization’s intended aim via incorporating SDPC into functional operations. Employees might opt to increase performance by offering the appropriate information to people at the appropriate time and under the appropriate conditions. The IMP is an essential instrument for firms’ workers to collaborate and ensure continuous growth across all organizational departments to improve SDPC.

### Theoretical and Practical Implications

This study’s findings provide important theoretical implications. *Firstly*, this study established a conceptual model depending on RBV theory, which provided several unexpected connections in response to a shortage of existing research in CRGI. This research is the pioneer study conducted in the manufacturing sector to demonstrate that IMP may assist in efficiently achieving and using information resources, streamlining processes, and increasing SDPCs and CRGI. *Secondly*, this work broadens our awareness of the critical role of all components of SDPC (environmental, social, and economic) in enhancing the CRGI. Owing to enhanced information sharing and implementation across stakeholders, firms may adjust their production processes via the adoption of SDPC and determine where and how trash might be utilized to create a by-product or mitigate its negative impact on the environment (Ding et al., 2019). *Thirdly*, our study quantified the mediation effect of SDPC, suggesting suitable recommendations for efficiency of cost and ecological deterioration for improving the green performance of firms. For instance, the worldwide adoption of hybrid-electric automobiles demonstrates that SDPC may transform a high-carbon sector into a greener, ecological, and cost-effective.

The study makes significant practical insights by endorsing the need for an internal IMP as a foundation for realizing the distinct benefits of SDPC within their operations to be more environmentally friendly. *Firstly*, policymakers should be alert and implement targeted training programs for personnel growth to evolve a culture of sustainability that adheres to the green strategic approach to increase profit and minimize the environmental effect. *Secondly*, although this research urges senior management and experts to incorporate SDPC, the efficient application requires acquisition, assimilation, and application of information to their processes. This study will aid in the development of an effective financial penalty and refund structure for manufacturers that breach applicable environmental legislation. Government regulators should give stakeholders tax breaks and low-interest loans to encourage them to incorporate sustainability initiatives into their processes. *Thirdly*, in light of the United Nations’ SDGs, conservationists and world leaders put enormous pressure on developing nations to enhance SDPC by integrating new and greener manufacturing technology. China has a chance to learn from the experiences of industrialized nations and implement remedial measures to avoid environmental deterioration caused by ineffective industrial activities. On the other side, the legislators should promote and successfully implement policies that foster a greener business climate and simplify things for businesses to transition away from fossil fuels and toward renewable energy sources (Irfan and Ahmad, 2022). This will increase the company’s understanding of environmental issues and foster CRGI.

Due to a lack of funding and time, this study contains limitations that may allow for further research. We employed a cross-sectional design for this investigation; however, a longitudinal design is recommended in the future to acquire more conclusive findings. We obtained data mostly from an emerging economy. Scholars are encouraged to reproduce this framework and expand this research to varied locations in the future to conduct a complete assessment of circular economy projects; such endeavors have not been a concern for global enterprises’ sustainable product creation. Additionally, comparative research is strongly needed to increase the generalization of this work. Our study has shown that IMP is necessary for forming SDPs and CGI. Finally, future studies may integrate other mediating or moderating factors, including green information sharing conduct, adsorption skills, and information transmission internally and externally related to sustainability aims.

## Data Availability Statement

The raw data supporting the conclusions of this article will be made available by the authors, without undue reservation.

## Ethics Statement

This study was reviewed and approved by the Institutional Review Board of North China Electric Power University, China (protocol code 642-8 on 12-01-2022) and according to the according to the Declaration of Helsinki guidelines. The patients/participants provided their written informed consent to participate in this study.

## Author Contributions

WH: writing – original draft, variable construction, and methodology. KC: supervision, funding acquisition and writing – review and editing. IK: writing – review and editing. NN: methodology and writing – review and editing. MI: conceptualization, software, methodology, formal analysis, data handling and writing – review and editing. AD: writing – review and editing. All authors contributed to the article and approved the submitted version.

## Conflict of Interest

The authors declare that the research was conducted in the absence of any commercial or financial relationships that could be construed as a potential conflict of interest.

## Publisher’s Note

All claims expressed in this article are solely those of the authors and do not necessarily represent those of their affiliated organizations, or those of the publisher, the editors and the reviewers. Any product that may be evaluated in this article, or claim that may be made by its manufacturer, is not guaranteed or endorsed by the publisher.

## References

[B1] AbbasJ. (2020). Impact of total quality management on corporate green performance through the mediating role of corporate social responsibility. *J. Clean. Prod.* 242:118458. 10.1016/j.jclepro.2019.118458

[B2] AbbasJ.SaǧsanM. (2019). Impact of knowledge management practices on green innovation and corporate sustainable development: a structural analysis. *J. Clean. Prod.* 229 611–620. 10.1016/j.jclepro.2019.05.024

[B3] AhmadB.DaL.AsifM. H.IrfanM.AliS. (2021). Understanding the antecedents and consequences of service-sales ambidexterity: a motivation-opportunity-ability (MOA) framework. *Sustainability* 13:9675. 10.3390/su13179675

[B4] AhmadB.IrfanM.SalemS.AsifM. H. (2022). Energy efficiency in the post-COVID-19 Era: exploring the determinants of energy-saving intentions and behaviors. *Front. Energy Res.* 9:824318. 10.3389/fenrg.2021.824318

[B5] AnH.RazzaqA.HaseebM.MihardjoL. W. W. (2021). The role of technology innovation and people’s connectivity in testing environmental Kuznets curve and pollution heaven hypotheses across the belt and road host countries: new evidence from method of moments quantile regression. *Environ. Sci. Pollut. Res.* 28 5254–5270. 10.1007/s11356-020-10775-3 32960444

[B6] AndersénJ. (2021). A relational natural-resource-based view on product innovation: the influence of green product innovation and green suppliers on differentiation advantage in small manufacturing firms. *Technovation* 104:102254. 10.1016/j.technovation.2021.102254

[B7] ArditoL.Messeni PetruzzelliA.PascucciF.PeruffoE. (2019). Inter-firm R&D collaborations and green innovation value: the role of family firms’ involvement and the moderating effects of proximity dimensions. *Bus. Strateg. Environ.* 28 185–197. 10.1002/bse.2248

[B8] AwanU.ArnoldM. G.GölgeciI. (2021). Enhancing green product and process innovation: towards an integrative framework of knowledge acquisition and environmental investment. *Bus. Strateg. Environ.* 30 1283–1295. 10.1002/bse.2684

[B9] BarneyJ. B. (2000). Firm resources and sustained competitive advantage. *Adv. Strateg. Manag.* 17 203–227. 10.1016/S0742-3322(00)17018-4

[B10] BarneyJ. B.KetchenD. J.WrightM. (2011). The future of resource-based theory: revitalization or decline? *J. Manag.* 37 1299–1315. 10.1177/0149206310391805

[B11] BhuttoT. A.FarooqR.TalwarS.AwanU.DhirA. (2021). Green inclusive leadership and green creativity in the tourism and hospitality sector: serial mediation of green psychological climate and work engagement. *J. Sustain. Tour.* 29 1716–1737. 10.1080/09669582.2020.1867864

[B12] ChangC. H. (2016). The determinants of green product innovation performance. *Corp. Soc. Responsib. Environ. Manag.* 23 65–76. 10.1002/csr.1361

[B13] ChenY. S.LaiS. B.WenC. T. (2006). The influence of green innovation performance on corporate advantage in Taiwan. *J. Bus. Ethics* 67 331–339. 10.1007/s10551-006-9025-5

[B14] CuiR.WangJ.XueY.LiangH. (2020). Interorganizational learning, green knowledge integration capability and green innovation. *Eur. J. Innov. Manag.* 24 1292–1314. 10.1108/EJIM-11-2019-0325

[B15] DarrochJ. (2005). Knowledge management, innovation and firm performance. *J. Knowl. Manag.* 9 101–115.

[B16] DavenportM.DelportM.BlignautJ. N.HichertT.van der BurghG. (2019). Combining theory and wisdom in pragmatic, scenario-based decision support for sustainable development. *J. Environ. Plan. Manag.* 62 692–716. 10.1080/09640568.2018.1428185

[B17] DingX.QuY.ShahzadM. (2019). The impact of environmental administrative penalties on the disclosure of environmental information. *Sustainbility* 11:5820. 10.3390/su11205820

[B18] ElkingtonJ. (1998). Partnerships from cannibals with forks: the triple bottom line of 21st-century business. *Environ. Qual. Manag.* 8 37–51. 10.1002/tqem.3310080106

[B19] FangZ.RazzaqA.MohsinM.IrfanM. (2022). Spatial spillovers and threshold effects of internet development and entrepreneurship on green innovation efficiency in China. *Technol. Soc.* 68:101844. 10.1016/j.techsoc.2021.101844

[B20] FieldA. (2013). *Discovering Statistics Using IBM SPSS Statistics.* Sage: Thousand Oaks, CA.

[B21] GengD.LaiK.ZhuQ. (2021). Eco-innovation and its role for performance improvement among Chinese small and medium-sized manufacturing enterprises. *Int. J. Prod. Econ.* 231:107869. 10.1016/j.ijpe.2020.107869

[B22] GrantR. M. (1997). The knowledge-based view of the firm: implications for management practice. *Long Range Plann.* 30 450–454. 10.1016/S0024-6301(97)00025-3

[B23] HairJ. F.Jr.MatthewsL. M.MatthewsR. L.SarstedtM. (2017). PLS-SEM or CB-SEM: updated guidelines on which method to use. *Int. J. Multivar. Data Anal.* 1:107. 10.1504/ijmda.2017.10008574 35009967

[B24] HaoY.DongX. Y.DengY. X.LiL. X.MaY. (2016). What influences personal purchases of new energy vehicles in China? An empirical study based on a survey of Chinese citizens. *J. Renew. Sustain. Energy* 8:065904. 10.1063/1.4966908

[B25] HertO. (1995). Corporate governance: some theory and implications. *Econ. J.* 105 678–689.

[B26] HojnikJ.RuzzierM. (2016). What drives eco-innovation? A review of an emerging literature. *Environ. Innov. Soc. Transitions* 19 31–41. 10.1016/j.eist.2015.09.006

[B27] HuangJ. W.LiY. H. (2017). Green innovation and performance: the view of organizational capability and social reciprocity. *J. Bus. Ethics* 145 309–324. 10.1007/s10551-015-2903-y

[B28] IrfanM.AhmadM. (2021). Relating consumers’ information and willingness to buy electric vehicles: does personality matter? *Transp. Res. Part D Transp. Environ.* 100:103049. 10.1016/j.trd.2021.103049

[B29] IrfanM.AhmadM. (2022). Modeling consumers’ information acquisition and 5G technology utilization: is personality relevant? *Pers. Individ. Differ.* 188:111450. 10.1016/j.paid.2021.111450

[B30] IrfanM.ElavarasanR. M.AhmadM.MohsinM.DagarV.HaoY. (2022). Prioritizing and overcoming biomass energy barriers: application of AHP and G-TOPSIS approaches. *Technol. Forecast. Soc. Change* 177:121524. 10.1016/j.techfore.2022.121524

[B31] IrfanM.HaoY.PanjwaniM. K.KhanD.ChandioA. A.LiH. (2020). Competitive assessment of South Asia’s wind power industry: SWOT analysis and value chain combined model. *Energy Strateg. Rev.* 32:100540. 10.1016/j.esr.2020.100540

[B32] IslamM. M.IrfanM.ShahbazM.VoX. V. (2021). Renewable and non-renewable energy consumption in Bangladesh: the relative influencing profiles of economic factors, urbanization, physical infrastructure and institutional quality. *Renew. Energy* 184 1130–1149. 10.1016/j.renene.2021.12.020

[B33] JinruL.ChangbiaoZ.AhmadB.IrfanM.NazirR. (2021). How do green financing and green logistics affect the circular economy in the pandemic situation: key mediating role of sustainable production. *Econ. Res. Istraz.* 1–21. 10.1080/1331677X.2021.2004437

[B34] KhanS. A. R.RazzaqA.YuZ.MillerS. (2021). Industry 4.0 and circular economy practices: a new era business strategies for environmental sustainability. *Bus. Strateg. Environ.* 30 4001–4014. 10.1002/bse.2853

[B35] LeeV. H.LeongL. Y.HewT. S.OoiK. B. (2013). Knowledge management: a key determinant in advancing technological innovation? *J. Knowl. Manag.* 17 848–872. 10.1108/JKM-08-2013-0315

[B36] LeguinaA. (2015). A primer on partial least squares structural equation modeling (PLS-SEM). *Int. J. Res. Method Educ.* 38 220–221. 10.1080/1743727x.2015.1005806

[B37] LiD.ZhengM.CaoC.ChenX.RenS.HuangM. (2017). The impact of legitimacy pressure and corporate profitability on green innovation: evidence from China top 100. *J. Clean. Prod.* 141 41–49. 10.1016/j.jclepro.2016.08.123

[B38] LimM. K.TsengM. L.TanK. H.BuiT. D. (2017). Knowledge management in sustainable supply chain management: improving performance through an interpretive structural modelling approach. *J. Clean. Prod.* 162 806–816. 10.1016/j.jclepro.2017.06.056

[B39] LucianettiL.Chiappetta JabbourC. J.GunasekaranA.LatanH. (2018). Contingency factors and complementary effects of adopting advanced manufacturing tools and managerial practices: effects on organizational measurement systems and firms’ performance. *Int. J. Prod. Econ.* 200 318–328. 10.1016/j.ijpe.2018.04.005

[B40] MillsA. M.SmithT. A. (2011). Knowledge management and organizational performance: a decomposed view. *J. Knowl. Manag.* 15 156–171. 10.1108/13673271111108756

[B41] NidumoluR.PrahaladC. K.RangaswamiM. R. (2009). Why sustainability is now the key driver of innovation. *Harv. Bus. Rev.* 57–64.

[B42] NunnallyJ. C. (1994). *Psychometric Theory 3E.* New York, NY: Tata McGraw-hill education.

[B43] OoiK. B. (2014). TQM: a facilitator to enhance knowledge management? A structural analysis. *Expert Syst. Appl.* 41 5167–5179.

[B44] RaufA.OzturkI.AhmadF.ShehzadK.ChandiaoA. A.IrfanM. (2021). Do Tourism development, energy consumption and transportation demolish sustainable environments? Evidence from Chinese Provinces. *Sustainability* 13:12361. 10.3390/su132212361

[B45] RehmanA.DeyuanZ.ChandioA. A.IrfanM. (2020). Does electricity production from different sources in Pakistan have dominant contribution to economic growth? Empirical evidence from long-run and short-run analysis. *Electr. J.* 33:106717. 10.1016/j.tej.2020.106717

[B46] ReuterK. E.SchaeferM. S. (2017). Illegal captive lemurs in Madagascar: comparing the use of online and in-person data collection methods. *Am. J. Primatol.* 79:22541. 10.1002/ajp.22541 26927567

[B47] SarkisJ.Gonzalez-TorreP.Adenso-DiazB. (2010). Stakeholder pressure and the adoption of environmental practices: the mediating effect of training. *J. Oper. Manag.* 28 163–176. 10.1016/j.jom.2009.10.001

[B48] SaunilaM.UkkoJ.RantalaT. (2018). Sustainability as a driver of green innovation investment and exploitation. *J. Clean. Prod.* 179 631–641. 10.1016/j.jclepro.2017.11.211

[B49] SavinoM. M.ShafiqM. (2018). An extensive study to assess the sustainability drivers of production performances using a resource-based view and contingency analysis. *J. Clean. Prod.* 204 744–752.

[B50] ShahN.SoomroB. A. (2021). Internal green integration and environmental performance: the predictive power of proactive environmental strategy, greening the supplier, and environmental collaboration with the supplier. *Bus. Strateg. Environ.* 30 1333–1344. 10.1002/bse.2687

[B51] ShahzadM.QuY.Ur RehmanS.ZafarA. U.DingX.AbbasJ. (2020a). Impact of knowledge absorptive capacity on corporate sustainability with mediating role of CSR: analysis from the Asian context. *J. Environ. Plan. Manag.* 63 148–174. 10.1080/09640568.2019.1575799

[B52] ShahzadM.QuY.ZafarA. U.RehmanS. U.IslamT. (2020c). Exploring the influence of knowledge management process on corporate sustainable performance through green innovation. *J. Knowl. Manag.* 24 2079–2106. 10.1186/s13054-016-1208-6 27885969PMC5493079

[B53] ShahzadM.QuY.ZafarA. U.DingX.RehmanS. U. (2020b). Translating stakeholders’ pressure into environmental practices – The mediating role of knowledge management. *J. Clean. Prod.* 275:124163.

[B54] ShahzadM.QuY.ZafarA. U.AppolloniA. (2021). Does the interaction between the knowledge management process and sustainable development practices boost corporate green innovation? *Bus. Strateg. Environ.* 30 4206–4222. 10.1002/bse.2865

[B55] SongM.YangM. X.ZengK. J.FengW. (2020). Green knowledge sharing, stakeholder pressure, absorptive capacity, and green innovation: evidence from Chinese manufacturing firms. *Bus. Strateg. Environ.* 29 1517–1531. 10.1002/bse.2450

[B56] SongW.YuH. (2018). Green innovation strategy and green innovation: the roles of green creativity and green organizational identity. *Corp. Soc. Responsib. Environ. Manag.* 25 135–150. 10.1002/csr.1445

[B57] TanveerA.ZengS.IrfanM. (2021). Do perceived risk, perception of self-efficacy, and openness to technology matter for solar PV adoption? An application of the extended theory of planned behavior. *Energies* 14:5008. 10.3390/en14165008

[B58] TsengM. L.LimM. K.WuK. J. (2018). Corporate sustainability performance improvement using an interrelationship hierarchical model approach. *Bus. Strateg. Environ.* 27 1334–1346. 10.1002/bse.2182

[B59] WangC. H. (2020). An environmental perspective extends market orientation: green innovation sustainability. *Bus. Strateg. Environ.* 29 3123–3134. 10.1002/bse.2561

[B60] WenC.AkramR.IrfanM.IqbalW.DagarV.Acevedo-DuquedÁ (2022). The asymmetric nexus between air pollution and COVID-19: evidence from a non-linear panel autoregressive distributed lag model. *Environ. Res.* 209:112848. 10.1016/j.envres.2022.112848 35101402PMC8800540

[B61] WestlandJ. C. (2010). Lower bounds on sample size in structural equation modeling. *Electron. Commer. Res. Appl.* 9 476–487. 10.1007/s11121-014-0489-8 24752569PMC4207737

[B62] WuH.BaN.RenS.XuL.ChaiJ.IrfanM. (2021). The impact of internet development on the health of Chinese residents: transmission mechanisms and empirical tests. *Socioecon. Plann. Sci.* 81:101178. 10.1016/j.seps.2021.101178

[B63] XueP.MakC. M.CheungH. D. (2014). The effects of daylighting and human behavior on luminous comfort in residential buildings: a questionnaire survey. *Build. Environ.* 81 51–59. 10.1016/j.buildenv.2014.06.011

[B64] YangC.HaoY.IrfanM. (2021). Energy consumption structural adjustment and carbon neutrality in the post-COVID-19 era. *Struct. Chang. Econ. Dyn.* 59 442–453. 10.1016/j.strueco.2021.06.017 35317307PMC8506069

[B65] YousafZ. (2021). Go for green: green innovation through green dynamic capabilities: accessing the mediating role of green practices and green value co-creation. *Environ. Sci. Pollut. Res.* 28 54863–54875. 10.1007/s11356-021-14343-1 34018115

[B66] YumeiH.IqbalW.IrfanM.FatimaA. (2021). The dynamics of public spending on sustainable green economy: role of technological innovation and industrial structure effects. *Environ. Sci. Pollut. Res.* 1:1. 10.1007/s11356-021-17407-4 34797541

[B67] ZhangY.SunJ.YangZ.WangY. (2020). Critical success factors of green innovation: technology, organization and environment readiness. *J. Clean. Prod.* 264:121701. 10.1016/j.jclepro.2020.121701

